The article "The Application of a Computer Monitoring System Using IoT Technology" was retracted in 2023. Reasons: signs of a paper mill; suspected computer-generated content; unreliable results or conclusions; concerns about the data.

# The Application of a Computer Monitoring System Using IoT Technology

**DOI:** 10.1155/2022/4033886

**Published:** 2022-06-06

**Authors:** Zhu Zhao, Qian Hu

**Affiliations:** ^1^Hunan Communication Polytechnic, College of Intelligent Transportation, Changsha 410132, Hunan, China; ^2^Central South University of Forestry & Technology, College of Logistics & Transportation, Changsha 410004, Hunan, China

## Abstract

Through the information exchange of the Internet of Things, resources in multiple fields can be integrated to provide users with more comprehensive, diverse, and high-quality services. The computer monitoring system can effectively improve the intelligence and networking of the office and is widely used in many industries. The application of Internet of Things technology can effectively improve the intelligence and networking of computer monitoring systems. The Internet of Things technology can realize the interaction between things and people, help the computer monitoring system to obtain the required information, and truly realize comprehensive monitoring. Based on this, this paper first introduces the basic technology of the Internet of Things technology and analyzes the main points of the computer monitoring technology based on the Internet of Things at this stage and then takes a computer monitoring system as the research object, and further analyzes the computer monitoring system based on the Internet of Things technology to help relevant personnel better apply IoT technology to computer monitoring systems.

## 1. Introduction

The IoT is a network in which everything can be connected together and is an effective extension of the Internet that enables the interconnection of people, machines and objects. The IoT is a product of the development of network technology, and the core foundation is the Internet, which is a way to exchange information and achieve intelligent identification, tracking, and monitoring of objects. The development of IoT involves three key points: sensor network, radio frequency identification technology, and terminal system framework. They are the main means to achieve the function of IoT application and an important component to form IoT.

IoT technology makes the computer monitoring system more and more intelligent. The reason a computer monitoring system can become a unified and independent system is very much related to the application of IoT technology; the application layer of IoT technology will help the computer monitoring system to realize the real-time condition monitoring of the target, which can intelligently judge the properties of the monitoring target. IoT technology will also keep the main module of the computer monitoring system, the warning module. At the same time, the computer monitoring system will also record the real-time operating condition of the monitored target to provide convenience for future problem handling.

The article "The Application of a Computer Monitoring System Using IoT Technology" was retracted in 2023. Reasons: signs of a paper mill; suspected computer-generated content; unreliable results or conclusions; concerns about the data.

Combined with the definition of IoT, it can be regarded as one of the application methods of a ubiquitous network to meet the demand for information interaction between different physical objects and provide more convenient and comprehensive services. With the deepening of IoT research, IoT technology presents a diversified development trend, covering key technologies such as cloud computing and radio frequency identification sensors, which promotes the intelligent development of objects and forms a unique IoT technology idea. In the construction of modern cities, IoT technology idea plays an important role in different fields and provides technical support for the construction of a smart society. The IoT technology applied in a computer monitoring system mainly has the following kinds.

SIP protocol is a control protocol, which is mainly used to establish a session to meet the multiparty monitoring requirements of the computer monitoring system. The application of SIP protocol mainly includes the following aspects. First, regarding the user agent, SIP protocol will build monitoring request information through the application of terminal equipment and then respond to the request through the agent, so as to achieve the intelligence of monitoring. Second, regarding the registration server, which is the database of IoT, the database is to be used to store many kinds of information about the server, the user can retrieve the required information in the database, and then, the registration server will process and send the information. Third, through the proxy server, the user can make inquiries, and it can also forward requests related to the computer monitoring system, thus increasing the speed of information transmission in the same area. Fourth, the redirection server transmits information from inside the monitoring system to the external area, thus enabling the operation between different hardware in the same server.

The RTP protocol is used in computer monitoring systems for real-time transmission, first using UDP for transmission services and then using the RTP protocol to guarantee the ability of end-to-end transmission. The RTP protocol has the advantage of being flexible so that programmers can write their own source code for computer monitoring systems according to their actual needs, thus realizing a variety of functions for monitoring.

AVS standard is an audio and video coding and decoding standard, which effectively simplifies the coding and decoding of IoT technology in computer monitoring system and largely reduces the complexity of coding and decoding. In the process of application, there are no algorithms with high complexity and difficulty, which saves a lot of space for computer monitoring system. Third, the method of macroblock prediction is chosen, which reduces the difficulty level of encoding and decoding, and improves the speed of encoding and decoding. Fourth, the use of four-tap filters effectively improves the operation speed of the computer monitoring system.

The article "The Application of a Computer Monitoring System Using IoT Technology" was retracted in 2023. Reasons: signs of a paper mill; suspected computer-generated content; unreliable results or conclusions; concerns about the data.

TMSDM6446 chip is a processing chip, mainly used for computer monitoring systems in the audio as well as video processing. The chip is divided into peripherals and control modules. For example, in the DSP subsystem, a video image processor, the processor will monitor the system's video processing area into eight spaces that can operate independently, through the SCR for peripheral devices and serial interfaces and other connections. This processing chip as the core of the monitoring system not only can improve the efficiency of audio as well as video processing but it also contains all the functions, such as the computer monitoring system storage module and decoding module.

## 2. Related Work

The construction of the IoT needs several technologies to coordinate and cooperate, and its key technologies include the radio frequency identification technology, which uses wireless radio frequency technology to collect tag information through readers and realize the effective interaction of item information [1].

The realization of radio frequency identification mainly depends on the radio signal. With the help of the radio signal, it can accurately identify the relevant information of the specified object [2]. RF identification technology is an important perception node of the IoT. Through the combination of multiple perception nodes, the technology can constitute a complete regional IoT structure, when the specified object enters the IoT RF signal coverage area, the specified object's unique electromagnetic signal can be captured in real-time, through the reception of the decoder for signal reception, and the electromagnetic signal will be transmitted to the processing equipment. The electromagnetic signal processing can be obtained after the relevant information collection [3, 4] and accurate data recognition, and can operate normally in the rain, snow, and foggy weather with high reliability [5].

Regarding the sensor technology, according to the item information collection needs, different types of sensors are installed in the items to collect various item [6]. In the whole IoT technology system, sensor technology mainly undertakes most of the information collection tasks and belongs to the foundation of IoT technology [7]. At this stage, sensor devices gradually tend to intelligent, accurate, miniaturized development, and sensor sensitivity is greatly improved. Hysteresis is optimized. When the detection of object status or parameter changes, the sensor technology can quickly grasp the state or parameter change information [8]. Sensor devices are mostly dependent on the wireless network arrangement, so it is not affected by the distribution of wired lines and has the advantage of flexible deployment and simple networking in the application [9].

The article "The Application of a Computer Monitoring System Using IoT Technology" was retracted in 2023. Reasons: signs of a paper mill; suspected computer-generated content; unreliable results or conclusions; concerns about the data.

Using cloud computing technology to build the IoT platform, the collected data information is integrated, and support is provided for the application of IoT [10]. With the development of technology, 5G technology is now commercially available to provide support for the popularity of IoT, further improving the information interaction rate in IoT and shortening the information transmission response time [11]. Each object within the IoT system has a unique information identification to facilitate the retrieval of data information, which is increasingly large data information. Therefore, an operation is carried to combine the actual situation to build the corresponding database, through cloud computing technology to build a resource center, so that data information within the IoT can be orderly applied [12, 13]. To ensure the effect of cloud computing, a powerful cloud computer needs to be set so that cloud computing technology in the IoT system can be fully effective [14, 15].

The main technical indicators of IoT today have seven major categories. The details are shown in Table 1.

For the computer monitoring system of the IoT, the dissemination and application of 5G network technology plays a certain optimization role and requires in-depth research and analysis by the personnel concerned [16, 17]. 5G network technology is an advanced mobile communication technology with the goal of increasing the transmission rate of data in mobile devices, reducing the delay in the process of network application, and lowering the input cost, thus increasing the system capacity and achieving an effective connection between devices connectivity between devices [18].

Currently, 5G networks are moving toward diversification, broadband, and integration [19]. Under the role of data traffic, with the expansion of 5G range, ultradense heterogeneous network becomes a key technology to improve data rate, which can realize the effective application of multiple wireless nodes and help the development of IOT-based computer monitoring system [20].

The article "The Application of a Computer Monitoring System Using IoT Technology" was retracted in 2023. Reasons: signs of a paper mill; suspected computer-generated content; unreliable results or conclusions; concerns about the data.

## 3. Methods

The constructed IoT monitoring system needs to have system security control function and application security function as well as data security function. The designed information platform is built with security management guarantee system, and firewall hardware technology is introduced to realize the network security protection. The system for the application security is designed to mainly ensure the security of system operation and host resources, through identity verification and authorization management, and to ensure that legitimate users can use the resources normally and avoid malicious attacks. In terms of data security management, technical and management measures are taken to achieve effective response and treatment of emergencies, and the system can be restored immediately in case of emergencies to avoid information loss.

In the specific construction of computer monitoring system, the application of IoT technology to carry out the design can effectively cope with the number of monitoring and management objects and the complexity of professionalism, through the unified modeling process and the construction of monitoring system. According to the business division, the functional modules of the monitoring system include the monitoring and control function module, data acquisition function module, and comprehensive processing function module. To build a standard management system and establish a monitoring platform, the system architecture is shown in Figure 1.

The execution process of our data acquisition system under the cloud is as follows: system power on, initialization of each module, system initialization check, and the autoaddressing flag bit to determine whether the video manager slave addresses need to be readdressed sequentially. When autoaddressing is not required, the node controller master reads the global unique ID code of each slave station from EEPROM, which is obtained and stored during the first operation, then obtains the global unique ID code of the slave station through Modbus communication polling, and compares the ID read in EEPROM with the ID code obtained in the slave station to see if it is consistent. If the ID code of the slave is not the same, the alarm of “slave ID code is abnormal” will be reported, and the device will be initialized successfully and ready for operation.

Figure 2 shows the initialization flowchart of the computer monitoring system. When the system is deployed or redeployed for the first time, the system initializes into the automatic addressing mode. In step 1, the master broadcasts the readdressing data frame to all slaves via Modbus, and when the slaves receive the broadcast, they automatically enter the addressing mode and monitor the SIG_ACK port level signal. In step 2, the master outputs a high level signal to slave 1 using CTL_ACK, and when slave 1 monitors the port level change, it sends a Modbus data frame with its own globally unique ID code to the master and changes its own slave number to temporary slave number 0x. The master receives the globally unique ID code from the slave, assigns the slave number in the order of the slave, binds the globally unique ID number to the slave number and stores it in the EEPROM memory, then sends the data frame with the assigned slave number to the slave at 0xFF, and waits for the slave to confirm the data frame. In step 4, the slave modifies and writes the new slave number into the power-down hold register, then writes the confirmation data frame, and raises the CTL_ACK port level. When all slave numbers are assigned, the system is initialized successfully and ready. The node module calls the check_inputStatus() function to poll the spindle status and save the data to the corresponding structure of the node module during the operation phase.

  Typedef struct.
  {
  uint32_trunsign;
  uint32_tinput;
  uint32_toutput;
  uint32_tshieldFlags;
  uint8_tslaveID[SLAVENUM][ID_LENGTH];
  uint32_tstartDelay;
  uint32_tmidwayRecoveryDelay;
  uint32_tscissorCount[SCISSORNUM];
  }USERPARAM;
  Typedef struct.
  {
  uint16_treSendTimeoutALARAM;
  uint8_tslaveNumberErr;
  uint16_tslaveID_Conflict;
  uint8_tautoAddrErr:1;
  }ALARAM;

Figure 3 shows the network diagram of the computer monitoring system sensor network, using Modbus communication protocol to form the sensor network. The video data are uploaded to the cloud server based on TCP/IP MQTT protocol. The communication protocol of IoT monitoring system mainly includes two parts, MQTT IoT protocol and HTTP hypertext transfer protocol.

The article "The Application of a Computer Monitoring System Using IoT Technology" was retracted in 2023. Reasons: signs of a paper mill; suspected computer-generated content; unreliable results or conclusions; concerns about the data.

The system's functional implementation is based on MQTT server, MySQL database, and Web server, deployed in Aliyun's Linux cloud server. The communication logic and interaction process are shown in Figure 4.

The MQTT server in the IoT monitoring system is responsible for subscribing and forwarding MQTT client messages and client rights management to prevent nonpermitted MQTT clients. The MQTT client in the IoT monitoring system is a subthread running within the Web server process and transfers it to the MySQL database or reads the database data and publishes it to the MQTT server and finally forwards it to the destination MQTT client terminal, as shown in Figure 5.

Web server: based on Django version 3.0.7, we use the MTV (model-template-views) development model, as shown in Figure 2. IoT monitoring system achieves the main functions: (1) Web server through Ajax technology polling real-time presentation of monitoring data to visualize the large screen; (2) online modification of editing parameters and call the MQTT client to access the MQTT IoT protocol network to achieve the next modified data or manually pull the terminal equipment monitoring parameters, equipment parameters, and other functions; (3) multiuser rights management, according to the differences in the positions of factory employees to give different web rights management.

Using the video terminal equipment arranged at each location, the images are captured in real time, and the collected data information is transmitted and applied for feedback. The processing process of video data information is as follows. ① Storage and application of data after data acquisition, as evidence or other passages: this requires the preparation of disk arrays of appropriate capacity to achieve the storage of large data. ② Use manual methods to keep an eye on the collected video data; the collected unknown images need to be processed in advance to realize the dynamic monitoring of the surveillance site. ③ Application of computer equipment or other equipment and the implementation of screen recognition and data processing, to achieve effective savings on human costs: the existing computer monitoring system is mainly video surveillance subsystem. Its common IoT control system, with a simple structure and large number of features, and the use of CAN bus achieve effective transmission of multiple video signals and send it to the central host to stay for use.

## 4. Case Study

To better illustrate the effectiveness of our designed IOT-based computer monitoring system, we have applied it to the field of highway monitoring for testing. The smart highway operation relies on a huge hardware and software foundation to achieve effective management of the operation of highway traffic facilities through the wide application of highway traffic information. In order to better perform the functions of the intelligent highway system, relevant researchers propose to use the monitoring technology to monitor the intelligent highway operation status in real time, grasp the highway traffic time distribution and spatial distribution, timely discover illegal operation behaviors such as speeding, overloading and illegal transportation on the highway, assist the highway traffic operation management department to take reasonable measures for unexpected events, and reduce the risk of intelligent highway operation. Because of more vehicles and infrastructure running on the highway, when the highway is in the peak period of vehicle driving, it is difficult to analyze the highway operation status, and it is difficult to realize the real-time monitoring of intelligent highway operation.

The article "The Application of a Computer Monitoring System Using IoT Technology" was retracted in 2023. Reasons: signs of a paper mill; suspected computer-generated content; unreliable results or conclusions; concerns about the data.

Highway operation information mainly includes road condition information, infrastructure information, and highway weather information. According to three kinds of information acquisition needs, choose the corresponding monitoring equipment to collect the information, as shown in Table 2.

Using the vehicle detector and the camera to collect the road condition information, set an electronic label inside the vehicle detector. When the vehicles travel on the highway pass through the vehicle detector, the electronic label will actively or passively send out the radio frequency signal *F* to the vehicle. The radio frequency signal reaches the vehicle and reflects back. The reflected signal *N* is received by the information receiving end, and the vehicle electronic label information is read by the built-in card reader of the vehicle detector, which will be uploaded. Transmitted to the wisdom highway system, the electronic label vehicle information is paired, so as to obtain the highway vehicle identity information *V*=[*F*, *N*]. In addition, the vehicle detector is equipped with a wireless probe, and the probe measures the time, speed, and vehicle spacing of the vehicle passing the probe when the vehicle is traveling on the highway. A 360° panoramic camera is used to obtain highway surveillance video information, which is installed above a highway traffic light with an LED light source so that the 360° panoramic camera can capture high-quality surveillance video data even in cloudy, foggy, or rainy environments.

The key to the collection of this information by monitoring equipment is the deployment of detection points. For highways with stable geological environment, a detection point is set every 500 m or 750 m; for highway sections with average geological stability, a detection point is set every 300 m or 350 m; for highway sections with very poor geological stability, a detection point is set every 150 m or 200 m. A roadbed detector and a slope detector are placed at the deployed detection points, and the foundation sinking speed and slope deformation speed are calculated according to the foundation and slope data, and the calculation formula is as follows:

(1) $$\begin{array}{c} \left\{\begin{array}{c} x=\frac{t_{1}-t_{2}}{l_{1}-l_{2}},\\ b=\frac{t_{1}-t_{2}}{h_{1}-h_{2}}, \end{array}\right. \end{array}$$

where *x* denotes the roadbed subsidence speed; *t*_1_ denotes the initial monitoring time; *t*_2_ denotes the current monitoring time; *l* denotes the initial value of roadbed; *l*_2_ denotes the current roadbed height; *b* denotes the road slope deformation speed; *h*_1_ denotes the initial road slope; *h*_2_ denotes the current road slope. Number each highway section and store the roadbed information and slope information of the highway into the corresponding numbered file [21–25].

The article "The Application of a Computer Monitoring System Using IoT Technology" was retracted in 2023. Reasons: signs of a paper mill; suspected computer-generated content; unreliable results or conclusions; concerns about the data.

Use the IoT technology to connect a variety of smart highway networks and monitoring equipment to realize the data transmission between monitoring equipment and the smart highway system. The communication framework is shown specifically in Figure 6.

To facilitate the subsequent analysis and calculation of intelligent highway operation status, the original data obtained by the monitoring equipment needs to be preprocessed, and the process is shown in Figure 7.

As shown in Figure 7, first, the smart highway operation data should be integrated and processed, and the data information should be integrated into a data collection according to different road sections and different time periods. The integrated operation information is converted and processed, and the code is used to represent the intelligent highway operation information, and its coding rules are shown in Table 3.

The wisdom highway operation data are converted according to the coding rules in Table 3 to give new attributes to the data. In order to avoid the influence of abnormal data on the analysis of wisdom highway operation status, the original data containing noisy data, incomplete data, invalid data, and data not related to wisdom highway operation monitoring are deleted to ensure data quality. The key of original data cleaning is to distinguish abnormal data. This time the quartile method is used to symmetrically clean the data, the upper and lower two quartiles of the upper and lower quartiles of wisdom highway operation data, that is, the upper and lower limits of the intelligent highway operation data cleaning, and the data beyond the limit is considered as abnormal data, which is expressed by the formula as follows.

(2) $$\begin{array}{c} \left\{\begin{array}{c} L_{\text{down}}=B-1.5\left(C-B\right),\\ L_{\text{up}}=B+1.5\left(C-B\right), \end{array}\right. \end{array}$$

In this formula, *L*_down_ represents the lower limit of the valid interval of the intelligent highway operation data; *B* represents the upper quantile of the intelligent highway operation data; *C* represents the lower quantile of the intelligent highway operation data; *L*_up_ represents the upper limit of the valid interval of the intelligent highway operation data. The previously mentioned formula is used to determine the interval range of the valid data, and the symmetry cleaning process is performed on the intelligent highway operation data according to the range, and finally, the dimensionality of the data is reduced and the space occupied by the data is reduced by statute processing of the data samples.

The article "The Application of a Computer Monitoring System Using IoT Technology" was retracted in 2023. Reasons: signs of a paper mill; suspected computer-generated content; unreliable results or conclusions; concerns about the data.

Based on this, the highway data is analyzed, and the current intelligent highway operation status is predicted. The factors affecting the operation status of smart highway mainly include road section congestion, visibility, road surface smoothness, and infrastructure safety, so the four factors are selected as the evaluation indexes of smart highway operation status, and the specific values of the four evaluation indexes are calculated by using the preprocessed data, among which the road section congestion is mainly related to the road flow, vehicle speed, and vehicle spacing, and its calculation formula is

(3) $$\begin{array}{c} O=\frac{W\cdot C\cdot T\cdot E}{L_{*}}, \end{array}$$

where *O* denotes the current congestion of the smart highway section; *W* denotes the value of vehicle flow on the highway road; *T* denotes the average distance between vehicles on the highway; *E* denotes the number of vehicles on the highway section; *L*_*∗*_ denotes the area of this smart highway section. The highway visibility is calculated based on the highway meteorological data with the following equation:

(4) $$\begin{array}{c} R=\sqrt{U\cdot K\cdot \frac{N}{Q}}. \end{array}$$

*R* denotes highway visibility; *U* denotes highway fogfall; *K* denotes highway snowfall; *N* denotes highway rainfall; *Q* denotes air density around the highway [26–30]. According to the deformation of highway slope and foundation subsidence, the safety of highway infrastructure is calculated as follows:

(5) $$\begin{array}{c} F=\frac{x\varphi +b\mu }{\psi }. \end{array}$$

*F* denotes the highway infrastructure safety degree; *φ* denotes the highway foundation sinking amount; *μ* denotes the highway slope deformation amount; *ψ* denotes the maximum tolerance limit of highway infrastructure damage. The smoothness of highway pavement is estimated according to the condition of highway pavement, and its calculation formula is

(6) $$\begin{array}{c} X=\left(Z+I+J\right)A, \end{array}$$

where *X* denotes the current pavement smoothness of the smart highway; *Z* denotes the snow volume of the highway pavement; *I* denotes the humidity of the highway pavement; *J* denotes the thickness of the ice layer of the highway pavement; *A* denotes the initial friction of the highway pavement. Based on the actual values of the four indicators, the operational state value of the smart highway is estimated, and its calculation formula is

(7) $$\begin{array}{c} \nu =\sum_{n=1}O\cdot R\cdot F\cdot X. \end{array}$$

*ν* indicates the operating status value of a section of the smart highway. The higher the operation status value means the better the operation status of the intelligent highway, and generally, the status value takes a range between −1 and 1, and the four levels are set. According to the different levels, the evaluation of the operation status of the smart highway is realized, and the reference basis is provided for the subsequent smart highway operation control.

The article "The Application of a Computer Monitoring System Using IoT Technology" was retracted in 2023. Reasons: signs of a paper mill; suspected computer-generated content; unreliable results or conclusions; concerns about the data.

By limiting the speed of highway vehicles and reducing the traffic flow of highway vehicles, the influence of four factors on the operation of smart highway, such as visibility, infrastructure safety, road surface smoothness, and congestion, is reduced, and the traffic flow of smart highway vehicles with state levels 1, 2 and 3 is controlled according to the previously mentioned analysis as shown in Table 4.

According to Table 4, the parameters of the speed limit value of vehicles on the intelligent highway are adjusted and optimized to control the traffic flow of the intelligent highway operation to complete the monitoring.

Taking a wisdom highway as the experiment object, the road length is 10000 m, the road width is 15 m, the roadbed height is 2.5 m, and the side slope angle is 26°. The experiment uses the design technology and traditional technology to monitor the operation status of the wisdom highway. The experiment divides the road into 10 sections; each section length is 1000 m. According to the actual situation of the road, a weather detector, two road sensors, two vehicle detectors, three 360° panoramic cameras, a roadbed detector, a side slope detector are installed in each section. The experiment monitored the 10 pavements for 30 days and obtained 123.15 GB of monitoring data, and the amount of monitoring data was 103.42 GB after data preprocessing, using the monitoring data to analyze the operation status of the intelligent highway as shown in Table 5.

According to the analysis of the operation status of the intelligent highway in Table 5, the highest level of the operation status of the highway is grade 3 and the lowest level is grade 1. The speed limit of the vehicle driving on the intelligent highway is determined as 40 km/h, and the average limit is 60 km/h. After the control, no traffic jam has occurred on the highway. This experiment takes the monitoring error as the technical performance evaluation index and uses software to calculate the technical monitoring error, as shown in Figures 8(a) and 8(b).

From the data in Figure 8, we can see that the designed computer monitoring error based on IoT technology is relatively small, the average monitoring error is 0.001, and the maximum monitoring error is only 0.003, which means that the designed technology has high accuracy. The maximum monitoring error of traditional technology can reach 0.864, and the average monitoring error is 0.468, which is much higher than the designed technology. Therefore, the experimental results prove that the design technology can better meet the operation monitoring accuracy requirements compared with the traditional technology.

The article "The Application of a Computer Monitoring System Using IoT Technology" was retracted in 2023. Reasons: signs of a paper mill; suspected computer-generated content; unreliable results or conclusions; concerns about the data.

## 5. Conclusion

In summary, the application of IoT technology has promoted the development of computer monitoring systems. An analysis can be drawn, and it can be seen through the experiments in this paper that the application of IoT technology can enable computer monitoring systems to achieve several functions, such as monitoring communication. The technical idea of forming multidomain fusion sharing and ubiquitous integrated services can be further considered later. Technicians should establish a sound technical system to build a wisdom monitoring system, according to the Internet of Things platform application scenarios, and clarify the functions of the wisdom monitoring system, applied to all aspects of the development of modern computer monitoring industry, to provide users with wisdom monitoring, and effectively play the advantages of Internet of Things technology.

## Figures and Tables

**Figure 1:** Architecture of the computer monitoring system.

**Figure 2:** MTV development model diagram.

**Figure 3:** Sensor network grouping diagram for under cloud system.

**Figure 4:** The initialization process of the system under the cloud.

**Figure 5:** IoT monitoring system composition diagram.

**Figure 6:** IoT-based intelligent highway operation data communication framework.

**Figure 7:** Schematic diagram of preprocessing of intelligent highway operation data.

**Figure 8:** (a) Comparison of different technical monitoring errors with our monitoring system. (b) Comparison of different technical monitoring errors with traditional monitoring system.

**Table 1:** Seven kinds of mainstream IoT main technical indicators.

IoT	Operating frequency band	Popular area	Transmission rate	Transmission distance(m)	Transmitting power (mW)	Application range
Bluetooth	2400∼2483.5 MHz	Global	1–24 Mbps	1–100	1–100	Point-to-point transmission of mouse, cell phone, computer, wireless headset, etc

ZigBee	2.4 GHz	Global	250 kbit/s			
	868 MHz	Europe	20 kbit/s	10–75(Addable relay)	1–100	Smart home; building automation; home automation
	915 MHz	United States	40 kbit/s			

Z-wave	908.42 MHz/868.42 MHz	USA/Europe	9.6 kbps/40 kbps	30(Indoor)-100(Outdoor)	1	Smart home; monitoring and control

SigFox	868 MHz/915 MHz	Europe/USA	100 bps	1–50000	<100	Remote meter reading, monitoring; smart home

WiFi	2.4 GHz/5 GHz	Global	1 Mbps to1 Gbps	50–100	<320	Wireless LAN

NB-IOT	Authorized toll bands below 1 GHz	Global	<100 kbps	1–20000	<100	Loop data collection and monitoring; positioning, home, bicycle

LoRa	433 MHz	Global				
	470∼510 MHz	China				
	780 MHz	China	0.3–50 kbps	1–20000	<100	Smart home; logistics eye tracking; smart building
	868 MHz	Europe				
	915 MHz	United States				

The article "The Application of a Computer Monitoring System Using IoT Technology" was retracted in 2023. Reasons: signs of a paper mill; suspected computer-generated content; unreliable results or conclusions; concerns about the data.

**Table 2:** Wisdom highway operation information acquisition.

Monitoring equipment type	Name	Function
Highway environmental safety monitoring equipment	Vehicle detectors	Get information on vehicle speed, traffic flow, workshop distance, etc.
	Weather detector	Get information on wind speed, wind direction, rainfall, snowfall, fog, etc.
	Road surface sensor	Get information of road ice, snow, humidity, etc.
	Environmental sensors	Obtain highway environmental visibility information

Highway structural safety monitoring equipment	Roadbed detector	Get highway roadbed information
	Side slope detector	Obtain highway slope information

Video surveillance equipment	Cameras	Obtain monitoring video information

**Table 3:** Intelligent highway operation data field coding rules table.

Data name	Field name
Vehicle travel speed	SDFSF_ETAF
Vehicle spacing	GDE_TWIOAQ
Highway vehicle flow	OOW_ERUAFS
Highway road snow accumulation	VHPMYG_QKSDF
Highway road surface humidity	PSH_DUKUAU
Road surface ice	VKOOA_WUHF
Highway roadbed	BAJL_PSFSY
Highway slope	ASYRQP_SHIF
Highway rainfall	OQ_OSGFHATR
Road snowfall	SOARQJP_HAQIR
Road fog	SGFHAU_HSIF
Road visibility	DNFA_JOJASF

**Table 4:** Traffic flow control standard of intelligent highway operation.

Operation level	Number of pavement lanes of smart highway			
	2	4	6	8
Level 1	30 Km/h	30 Km/h	40 Km/h	40 Km/h
Level 2	40 Km/h	40 Km/h	60 Km/h	60 Km/h
Level 3	60 Km/h	60 Km/h	80 Km/h	80 Km/h

**Table 5:** Analysis of wisdom highway operation status.

Monitoring time	Visibility	Smoothness	Safety	Crowdedness
6:30	0.265	0.595	0.485	0.865
12:30	0.268	0.488	0.698	0.638
18:30	0.167	0.695	0.755	0.259
22:30	0.369	0.528	0.595	0.947
27:30	0.295	0.287	0.372	0.268
32:30	0.365	0.269	0.285	0.359
35:30	0.582	0.377	0.345	0.282

## Data Availability

The experimental data used to support the findings of this study are available from the corresponding author upon request.
